The article "Adenylate Cyclase Toxin Tinkering With Monocyte-Macrophage Differentiation" was published in 2020. Journal: Front Immunol.

# Adenylate Cyclase Toxin Tinkering With Monocyte-Macrophage Differentiation

**DOI:** 10.3389/fimmu.2020.02181

**Published:** 2020-09-11

**Authors:** Jawid Nazir Ahmad, Peter Sebo

**Affiliations:** Laboratory of Molecular Biology of Bacterial Pathogens, Institute of Microbiology of the CAS, Prague, Czechia

**Keywords:** dedifferentiation, *Bordetella pertussis*, adenylate cyclase toxin, macrophages, monocytes

## Abstract

Circulating inflammatory monocytes are attracted to infected mucosa and differentiate into macrophage or dendritic cells endowed with enhanced bactericidal and antigen presenting capacities. In this brief Perspective we discuss the newly emerging insight into how the cAMP signaling capacity of *Bordetella pertussis* adenylate cyclase toxin manipulates the differentiation of monocytes and trigger dedifferentiation of the alveolar macrophages to facilitate bacterial colonization of human airways.

## Introduction

To proliferate at sufficient numbers on mucosal surfaces and transmit to a new host, bacterial pathogens have to evade host innate and adaptive immune responses (1). Host cells sense the microbe-associated molecular patterns (MAMPs) through an array of cell surface and intracellular sensors (e.g., TLRs and NOD-like receptors and other) and release cytokine and chemokine signals that attract circulating leukocytes, like neutrophils and monocytes, to the infected site (2). Growth factors and cytokines, such as M-CSF, GM-CSF, IL-4, type I interferons, and other signaling molecules produced in the tissue then shape the transition of infiltrating monocytes into macrophage or dendritic cells (DCs) (3–6). Differentiation of infiltrating monocytes at the mucosal surface involves several complex transition stages that lead to acquisition of macrophage capabilities involved in clearance of pathogens (7–9). The differentiated monocyte-derived cells are endowed with enhanced phagocytic and bactericidal capacities and contribute to initiation and shaping of adaptive B and T lymphocyte immune responses through presentation of antigens to T cells and cytokine release (3, 10).

The Gram-negative coccobacillus *Bordetella pertussis* is an obligate human pathogen that causes the respiratory illness called pertussis, or whooping cough. Newborns and infants are at a particular risk of a fatal course of pertussis due to a congenital immunosuppressive environment at their mucosa that limits the innate immune defenses (11). In fact, pertussis used to be the first cause of infant mortality in industrialized countries prior to introduction of efficient pertussis vaccines (12). Despite global vaccine coverage, the whooping cough illness remains the least-controlled vaccine-preventable infectious disease with estimated over 20 million cases and more than 150,000 deaths occurring annually world-wide (13). This is due to an amazing capacity of the pathogen to overcome the innate and adaptive immune defenses of host airway mucosa. If not complicated by a secondary infection, whooping cough is the only major infectious disease that is not accompanied by fever. It starts by a catarrhal phase with symptoms resembling the common cold, with runny nose, sneezing and cough that make *B. pertussis* infections highly contagious (14). *B. pertussis* bacteria employ a whole array of sophisticated virulence factors to subvert host immunity and convert the nasopharynx of the infected individual to a safe niche for proliferation to the high numbers and eliciting of catarrh needed for transmission by aerosol. The bacteria adhere to the ciliated epithelial cells of the upper airways through their fimbriae (FIM2/3), form microcolonies growing between the cilia of epithelial cells and eventually form a biofilm on ciliated epithelia (15, 16). The filamentous hemagglutinin (FhaB, processed to FHA), the outer membrane autotransporter pertactin (Prn) and tracheal colonization factor A (TcfA) mediate tight adhesion to epithelial and/or immune cell membrane and the Vag8, BrkA, and FHA proteins effectively inhibit bactericidal complement deposition on bacterial outer surface (16). Additional outer membrane autotransporters likely play as yet unknown roles in immune subversion by the bacterium and a Type Three Secretion System (T3SS) injectosome delivers the BteA/BopC effector into host cells to suppress inflammatory signaling by an as yet unknown mechanism (17, 18). Finally, *B. pertussis* secretes two major immunomodulatory protein toxins that manipulate signaling of host immune cells. The more notoriously known pertussis toxin (PT) is an AB_5_ family toxin that delivers into a broad variety of cell types an ADP-ribosylating enzyme (19). Its action inactivates the inhibitory Gα_i/o_ subunits of trimeric G proteins and thereby hijacks a whole array of G protein-coupled receptor (GPCR) signaling-regulated pathways (20). This accounts for the systemic effects of PT action, such as the delay in neutrophil arrival to the infected site due to inhibition of chemokine receptor expression, proliferation of lymphocytes and the leukocyte egress from bone marrow. It yields a potentially life-threatening hyperleukocytosis (21) with formation of mixed leukocyte aggregates in arterioles contributes to pulmonary hypertension and heart failure in infants (22). Perturbations of immune functions of lymphocytes by PT action are among other due to upregulated endogenous adenylyl cyclase activity and cAMP accumulation in PT-affected cells (21).

The other major toxin, the adenylate cyclase toxin-hemolysin (CyaA, ACT of AC-Hly) is a highly active cell invasive adenylyl cyclase enzyme on its own and belongs to the most potent factors by which *B. pertussis* disarms the innate immune system and hijacks the adaptive immune responses. At the local concentrations of CyaA produced on infected epithelial layers (23, 24) the toxin could act directly also on airway epithelial cells. CyaA can compromise the epithelial barrier function by cAMP signaling-triggered disruption of tight junctions between epithelial cells and can suppress antimicrobial peptide production (25). The toxin then would primarily target the sentinel cells of innate immunity through binding of complement receptor-3 (CR3, known as the α_M_β_2_ integrin or CD11b/CD18). CR3 is expressed on neutrophils, NK cells, monocytes, macrophages, dendritic cells and certain B cell subtypes (26–28). Upon engagement of the CD11b subunit of CR3, the CyaA toxin inserts into the plasma membrane of phagocytes and translocates into their cytosol its N-terminal adenylyl cyclase enzyme domain (29). This gets activated by binding of intracellular calmodulin and catalyzes a massive and unregulated conversion of cellular ATP into the key second messenger signaling molecule cAMP that ablates the bactericidal capacities of phagocytes (28, 30, 31). Signaling of cAMP near-instantly blocks Syk, RhoA and MAPK (e.g., p38 and ERK1/2) activities, thus inhibiting opsonophagocytic uptake of bacteria and the assembly of the NADPH oxidase, thereby blocking oxidative burst of neutrophils and preventing killing of bacteria by reactive oxygen species (32–34). At the same time cAMP signaling activates the tyrosine phosphatase SHP-1 and triggers AP-1 transcription factor dephosphorylation thereby blocking iNOS expression and inducible NO production by macrophages (35).

While not having been reported to exert systemic effects, the local CyaA action most likely delays or subverts also induction of adaptive T and B cell-mediated immune responses at the infected mucosa. Through its subversive cAMP signaling activity on CR3-expressing intraepithelial and submucosal dendritic cells (DC), the CyaA-mediated elevation of cAMP would deregulate DC maturation in response to TLR ligands. CyaA action blocks proinflammatory IL-12 and TNFα cytokine secretion and upregulates IL-10 release, while impairing the capacity of DCs to traffic, process and present antigens on MHC class II and I molecules to CD4^+^ and CD8^+^ T cells (36). At the same time, cAMP signaling enhances the migratory capacity of such tolerogenic DCs that are capable of expanding CD4^+^CD25^+^Foxp3^+^ T regulatory cells, limiting Th1 and eventually enhancing Th17 cell expansion (36–38). The biased cytokine secretion profile of T cells likely skews and/or delays also antibody response and this aspect of CyaA action still awaits exploration.

## *Bordetella pertussis* Adenylate Cyclase Toxin Subverts Monocyte Differentiation and Dedifferentiates Airway Macrophages to Less Bactericidal Monocyte-Like Cell Type

Recently, we observed that in *B. pertussis*-infected mouse lungs the CyaA toxin action inhibited differentiation of infiltrating monocytes into macrophage and dendritic cells (39). Due to its extremely high catalytic activity, CyaA at even very low amounts generates enough intracellular cAMP to elicit a subversive “signaling storm” in host phagocytes through activation of the protein kinase A (PKA)-directed pathways. Exposure to as little as 22.5 pM (4 ng/mL) CyaA provokes a complete inhibition of the M-CSF-driven transition of human monocytes into macrophages without affecting their viability and toxin concentrations over 50 pM (10 ng/mL) trigger apoptosis of human monocyte/macrophage cells (40–42).

Tissue-infiltrating monocytes are short-lived, lack the self-renewal ability and exhibit a modest phagocytic and bactericidal activity. In contrast, the more phagocytic and highly bactericidal mature macrophages are capable of self-renewal (6). We observed that exposure of monocytes to CyaA/cAMP signaling blocked M-CSF-driven formation of intracellular granules and prevented development of larger Golgi bodies and the formation of an expanded ER network typical for the mature macrophage cells (6, 42–44). Hence, CyaA/cAMP-elicited signaling restricted development of organelles required for enhanced synthesis and secretion of cytokines and providing membranes for formation of phagosomes (45–47). The mechanism by which CyaA-elicited cAMP signaling through the PKA-regulated pathways blocks M-CSF-triggered differentiation into macrophages requires further investigation. A plausible hypothesis would be that cAMP signaling inhibits the expression of the receptor for IL-2 (IL-2R) and thus reduced IL-2 signaling downregulates expression of the M-CSF receptor, making the CyaA-exposed monocytes insensitive to pro-differentiating signals (42, 48, 49).

Moreover, we observed that cAMP signaling of CyaA also provoked de-differentiation of mature terminally differentiated tissue-resident human alveolar macrophages back into monocyte-like cells (42). This likely plays a major role in immune evasion by the whooping cough agent. Dedifferentiation of macrophages to monocyte-like cells would relieve also the bactericidal pressure of the complement system, since macrophages contribute to host defense through production of complement components on the mucosa and by complement-dependent opsonophagocytic killing of bacteria (50, 51). With their self-renewal capacity, macrophages belong to the longest living immune cell types that patrol the airway mucosa (6). Lung alveoli harbor high numbers of tissue resident alveolar macrophages established during embryonic development. The CyaA-elicited macrophage cell shrinkage and loss of intracellular organelle number and size in primary human alveolar macrophages could plausibly be due to a cAMP/PKA-driven block of cell growth signaling emanating from the AKT/PKB and Hippo signaling pathways (41, 42, 52). Indeed, LATS1/2 phosphorylates and inactivates the downstream transcriptional regulator Yap/Taz that regulates expression of genes involved in cell size and organ growth (53). Upon phosphorylation by LATS1/2, Yap/Taz is sequestered by the 14-3-3 binding protein and degraded in the cytoplasm (54). Activation of PKA by CyaA-produced cAMP inhibits Syk signaling and RhoA (27, 32, 55) and inactivation of RhoA by PKA is known to induce LATS1/2 activity (56). Hence, it will be important to assess, if CyaA/cAMP signaling through PKA triggers an inhibitory phosphorylation of Yap on Ser^380^ by LATS1/2 (52). Through Yap-inactivating effects, the CyaA-generated cAMP signaling would inhibit cell size growth during both differentiation and dedifferentiation of macrophages (42, 52). This would possibly also delay the induction of adaptive immune responses, since macrophages are the prime source of IL-1β and IL-12 cytokines involved in CD4^+^ T-cell activation and expansion (57). The related *Bordetella bronchiseptica* bacteria were shown to reach the nose and lung-draining lymph nodes (58) and it deserves to be determined if the produced CyaA triggers de-differentiation of the macrophages at the sub-capsular sinus (SCS) of the lymph nodes (59). Preventing these cells from collecting particulate antigens and making these available to follicular B cells would compromise the induction of humoral immune response (59), possibly contributing to the chronic nature of *B. bronchiseptica* infections of mammals.

## Concluding Remarks

The bactericidal and antigen presenting capacities of macrophage and dendritic cells play a sentinel role in innate host defense and in induction of adaptive immune responses to bacterial infection. The respiratory pathogen *B. pertussis* utilizes a cAMP elevating toxin (CyaA) to reduce macrophage activities through a complex signaling network (schematically depicted in Figure 1 and in Figure 2) that inhibits monocyte differentiation into macrophage cells and triggers dedifferentiation of airway macrophages to the less phagocytic immune cell types. All these complex events would then compromise host's anti-*Bordetella* immune responses, enabling immune evasion and bacterial proliferation at the nasopharyngeal mucosa.

**Figure 1:** CyaA manipulates phagocyte differentiation. Monocytes get recruited to the infected tissue by the secreted chemoattractants and mature into macrophages. *B. pertussis* secreted CyaA and in part pertussis toxin action blocks the differentiation of monocytes into macrophage cells and provokes de-differentiation of patrolling alveolar human macrophages to less bactericidal monocyte-like cells.

**Figure 2:** Model for *B. pertussis* CyaA regulated complex signaling pathways to block the monocyte differentiation and to trigger macrophage dedifferentiation. CyaA toxin recognizes CD11b molecule on phagocytes to translocate its adenylate cyclase (AC) domain across the cell membrane. Upon interaction with the host cell protein calmodulin, AC enzyme gets activated and catalyzes the conversion of cellular ATP to cAMP. cAMP signal transduction via PKA then inactivates RhoA and/OR activates LATS1/2 to inhibit Yap regulated gene expression and prevents monocytes from acquiring bigger cell size, a typical macrophage feature; this signaling pathway could also block the macrophages from retaining large cell size and triggers their dedifferentiation. The decrease in Yap activity is paralleled by the inactivation of AKT/PKB to suppress the cell growth signaling in order to reduce cell size. Elevated cAMP level subverts IL-2 receptor signaling which upregulates the M-CSF receptor expression and that makes the monocyte less sensitive to pro-differentiating M-CSF growth factor. These complex CyaA-mediated signaling events culminate in subverting macrophage-based host protective functions to compromise the anti-*Bordetella* host immune responses.

## Data Availability Statement

The original contributions presented in the study are included in the article/supplementary material, further inquiries can be directed to the corresponding author/s.

## Author Contributions

JA conceived the paper and wrote the original draft. PS and JA modified the original text and prepared the final draft. All authors contributed to the article and approved the submitted version.

## Conflict of Interest

PS is co-inventors on several patents protecting CyaA as antigen for pertussis vaccines, PS is co-owner of the start-up company Revabiotech SE that aims at development of a next generation of whole-cell pertussis vaccine. The remaining author declares that the research was conducted in the absence of any commercial or financial relationships that could be construed as a potential conflict of interest.
